The article "IL-2 augments the sorafenib-induced apoptosis in liver cancer by promoting mitochondrial fission and activating the JNK/TAZ pathway" was retracted in 2019. Reasons: plagiarism; overlap with other authors' work.

# IL-2 augments the sorafenib-induced apoptosis in liver cancer by promoting mitochondrial fission and activating the JNK/TAZ pathway

**DOI:** 10.1186/s12935-018-0671-3

**Published:** 2018-11-09

**Authors:** Xiaoyan Ding, Wei Sun, Jinglong Chen

**Affiliations:** Cancer Center, Beijing Ditan Hospital, Capital Medical University, No 8, Jingshundong Street Chaoyang District, Beijing, 100015 China

**Keywords:** IL-2, Sorafenib, Mitochondrial fission, Liver cancer, JNK-TAZ pathways

## Abstract

**Background:**

Sorafenib is the standard targeted drug used to treat hepatocellular carcinoma (HCC), but the therapeutic response between individuals varies markedly. Recently, cytokine-based immunotherapy has been a topic of intense discussion in the fight against cancer. The aim of this study was to explore whether cytokine IL-2 could augment the anti-tumour effects of sorafenib on HCC.

**Methods:**

HepG2 and Huh7 cells were co-treated with sorafenib and IL-2 in vitro, and cellular viability and death were analysed through the MTT assay, TUNEL staining, LDH release assay, and western blotting. Mitochondrial function was measured via ELISA, immunofluorescence, and western blotting. Pathway blockers were used to establish the role of the JNK-TAZ pathways in regulating cancer cell phenotypes.

**Results:**

Our data demonstrated that sorafenib treatment increased the HCC apoptotic rate, repressed cell proliferation, and inhibited migratory responses, and these effects were enhanced by IL-2 supplementation. Mechanistically, the combination of IL-2 and sorafenib interrupted mitochondrial energy metabolism by downregulating mitochondrial respiratory proteins. In addition, IL-2 and sorafenib co-treatment promoted mitochondrial dysfunction, as evidenced by the decreased mitochondrial potential, elevated mitochondrial ROS production, increased leakage of mitochondrial pro-apoptotic factors, and activation of the mitochondrial death pathway. A molecular investigation revealed that mitochondrial fission was required for the IL-2/sorafenib-mediated mitochondrial dysfunction. Mitochondrial fission was triggered by sorafenib and was largely amplified by IL-2 supplementation. Finally, we found that IL-2/sorafenib regulated mitochondrial fission via the JNK-TAZ pathways; blockade of the JNK-TAZ pathways abrogated the inhibitory effects of L-2/sorafenib on cancer survival, growth and mobility.

**Conclusions:**

Altogether, these data strongly suggest that additional supplementation with IL-2 enhances the anti-tumour activity of sorafenib by promoting the JNK-TAZ-mitochondrial fission axis. This finding will pave the way for new treatment modalities to control HCC progression by optimizing sorafenib-based therapy.

**Electronic supplementary material:**

The online version of this article (10.1186/s12935-018-0671-3) contains supplementary material, which is available to authorized users.

## Background

Hepatocellular carcinoma (HCC), the sixth most common cancer worldwide, accounts for ~ 5.7% of the overall incidence of cancer [1]. Several risk factors have been associated with the development of HCC, including (but not limited to) hepatitis B infection, alcohol consumption, diabetes mellitus and smoking [2]. Despite advancements in uncovering the molecular aetiology of HCC, treatments for HCC are still unsatisfactory; the 5-year survival rate remains approximately 26% in patients receiving standard chemotherapy and/or radiotherapy [3].

Targeted therapy has been tested in several clinical trials and has been proven to provide a survival advantage for patients with HCC. Sorafenib is the first approved targeted therapy drug and is also the first-line FDA-approved tyrosine kinase inhibitor, improving the median overall survival time from 7.9 to 10.7 months in patients with HCC [4]. At the molecular level, sorafenib represses Raf kinase, a key protein mediating cancer proliferation [5]. Sorafenib also suppresses angiogenesis by modulating the Ras/Raf/MEK/ERK signalling pathway and VEGFR [6]. Notably, the tolerance and efficacy of sorafenib in Child–Pugh B patients have not been determined, and several reports argue that sorafenib does not seem to be an option for these patients [7]. Furthermore, the clinical benefit of sorafenib treatment is limited to an overall increase in survival time of 3 months [8]. Thus, these data indicate the therapeutic potential of sorafenib against the progression of HCC but suggest that it is also clinically necessary to optimize sorafenib-based treatment by combining it with other therapeutic strategies, such as immunotherapy.

Immunotherapy has demonstrated great promise in specifically killing cancer cells by multiple mechanisms [9]. Cytokine-based immunotherapy is currently a topic of intense discussion in the fight against cancer [10]. For example, supplementation with IL-7 has been found to repress the progression of acute lymphoblastic leukaemia [11], and in pancreatic cancer, the inhibition of IL-6 suppresses the metastatic invasion and migration of tumours [12]. Moreover, the regulation of CXCL13 modifies breast cancer cell viability via the CXCR5/ERK pathway [13]. In animal studies and cell experiments on liver cancer, the cytokine IL-2 has been documented to be a potential therapeutic target to limit tumour growth [14, 15]. In a clinical trial with small sample sizes, administration of IL-2 was found to play a beneficial role in suppressing the development and progression of HCC [16]. This finding was also supported by a previous study in which an IL-2 vaccine mediated the regression of HCC in mice [15]. As there is strong evidence supporting the suppressive effects of IL-2-based therapy against HCC progression, it is worthwhile to explore whether IL-2, in combination with sorafenib, can further reduce the proliferation of liver cancer cells.

Mitochondrial fission, which initiates the mitochondrial apoptosis pathway, is an early hallmark of cancer cell death [17, 18]. Excessive mitochondrial fission disrupts mitochondrial energy metabolism, evokes oxidative stress, causes cellular calcium overload, and promotes the activation of pro-apoptotic factors [19, 20]. Several attempts have been made to induce the activation of mitochondrial fission in various tumours such as those in pancreatic cancer [21], endometriosis [22], and breast cancer [23]. Based on the data gained from these studies, we wanted to determine whether IL-2 could augment sorafenib-mediated HCC apoptosis by activating mitochondrial fission. The JNK and TAZ pathways are the primary upstream regulators for mitochondrial fission in liver cancer and in breast cancer [24, 25]; however, whether IL-2 is capable of modifying mitochondrial fission via the JNK-TAZ axis has remained unknown. Thus, the aim of our study was to explore the efficacy of IL-2 in combination with sorafenib on inducing HCC apoptosis, with a focus on mitochondrial fission and the JNK-TAZ pathways.

## Materials and methods

### Cell culture and treatment

The HepG2 liver cancer cell line was purchased from the American Type Culture Collection (ATCC^®^ HB-8065™). The Huh7 liver cancer cell line and L02 normal liver cell line were purchased from the Cell Bank of the Chinese Academy of Sciences. The HepG2 and Huh7 cells were cultured in DMEM medium (#12800-017, Gibco) with 10% FBS (#10437-028, Gibco) at 37 °C/5% CO_2_. To induce damage, the cancer cells were treated with sorafenib (5 μM) for approximately 12 h. Another group of cells was treated with IL-2 (0–20 ng/ml) for 12 h according to a previous study [16]. To inhibit the activity of the JNK pathway, cells were treated with SP600125 (SP, 10 μM, Selleck Chemicals) 2 h before sorafenib/IL-2 treatment [26].

### Cellular viability and death evaluation

Cellular viability was measured with MTT and LDH release assays. The MTT assay was performed according to the methods used in a previous study [27]. Cells were plated onto a 96-well plate with the IL-2 and sorafenib treatment. MTT solution (Beyotime, China, Cat. No. C0009) was then added into the medium, and the cells were incubated for approximately 2 h at 37 °C/5% CO_2_. The optical density (OD) of the MTT solution was recorded using a microplate reader (490 nm absorbance; Epoch 2; BioTek Instruments, Inc., Winooski, VT, USA). An LDH release assay was conducted using a commercial kit (Beyotime, China, Cat. No. C0016) according to the manufacturer’s instructions [28].

Cellular death was measured via a TUNEL assay and the measurement of caspase-3 activity. TUNEL staining was performed using a One Step TUNEL Apoptosis Assay Kit (Beyotime, China, Cat. No. C1086) according to the manufacturer’s instructions. Caspase-3 activity was estimated using the Caspase 3 Activity Assay Kit (Beyotime, China, Cat. No. C1115), and the relative caspase-3 activity was measured compared to that of the control group using a microplate reader (430 nm absorbance; Epoch 2; BioTek Instruments, Inc., Winooski, VT, USA) [29].

### Oxidative stress measurement

Cellular oxidative stress was determined via ELISA as described in a previous study. Cells were washed with PBS and lysed using RIPA Lysis Buffer (Beyotime, China, Cat. No. P0013C). Then, the proteins were collected through high-speed centrifugation, and the concentrations of GSH (Beyotime, China, Cat. No. S0073), SOD (Beyotime, China, Cat. No. S0086) and GPX (Beyotime, China, Cat. No. S0058) were measured using commercial kits according to the manufacturers’ instructions [30].

### EdU staining and transwell assay

To analyse the cellular proliferation, EdU staining was conducted using the BeyoClick™ EdU Cell Proliferation Kit with Alexa Fluor 594 (Beyotime, China, Cat. No. C00788L). Cells were first washed with PBS. Fresh DMEM was then added, and 10 μM EdU was added into the medium. The cells were incubated for 2 h at 37 °C/5% CO_2_. After the incubation, the cells were again washed with PBS to remove the DMEM and the free EdU probe. The cells were then fixed in 4% paraformaldehyde at room temperature for 30 min before being stained with DAPI for 3 min. After an additional wash in PBS, the cells were observed under an inverted microscope [31].

A transwell assay was carried out to observe the cell migration response based on the methods of a previous study [32]. Cells at a density of 1 × 10^3^ were added into the upper chamber. DMEM with 2% FBS was loaded into the lower chamber. Subsequently, the cells were cultured at 37 °C/5% CO_2_ for 12 h. After the culture period, the non-migrated cells were removed, and the migrated cells were fixed with 3.7% paraformaldehyde for 30 min at room temperature. The migrated cells were then stained with 0.05% crystal violet for 15 min at room temperature in the dark. The number of migrated cells was recorded, and images were captured under an inverted microscope.

### Mitochondrial function detection

Mitochondrial function was measured by analysing the mitochondrial membrane potential, the mitochondrial permeability transition pore (mPTP) opening rate and the mitochondrial ROS generation. The mitochondrial membrane potential was determined by JC-1 staining [33]. Live cells were washed with PBS, and a JC-1 solution was then added to the medium. The cells were incubated at 37 °C/5% CO_2_ for 30 min, washed with PBS, loaded with DAPI, and then observed under a fluorescence microscope. The mPTP opening rate was recorded as described by a previous study. Cells were first washed with PBS and incubated with calcein-AM/cobalt at 37 °C/5% CO_2_ for 30 min. The cells were then washed with PBS again to remove the free probe. The optical density (OD) was recorded using a microplate reader (540 nm absorbance; Epoch 2; BioTek Instruments, Inc., Winooski, VT, USA). The mPTP opening rate was expressed relative to that of the control group [34]. Mitochondrial ROS production was measured via flow cytometry as described by a previous study. Cells were washed three times in PBS and incubated with MitoSOX Red Mitochondrial Superoxide Indicator (Molecular Probes, USA) for 30 min at 37 °C/5% CO_2_ in the dark. After incubation, the cells were washed three times in PBS at room temperature, and the mitochondrial ROS production was measured via flow cytometry [35].

### Western blotting

Cells were lysed in RIPA Lysis Buffer (Beyotime, China, Cat. No. P0013C). After high-speed centrifugation, the proteins were collected and quantified with the Enhanced BCA Protein Assay Kit (Beyotime, China, Cat. No. P0009). Subsequently, 40–60 μg of protein was loaded onto 10% SDS-PAGE gels and transferred to PVDF membranes. The membranes were washed with TBST and then blocked with 5% non-fat milk for 45 min at room temperature [36]. The membranes were then incubated at 4 °C overnight with the primary antibodies [CXCR4 (1:1000, Abcam, #ab1670), CXCR7 (1:1000, Abcam, #ab38089), cyclin D1 (1:1000, Abcam, #ab134175), PCNA (1:1000, Abcam, #ab18197), CDK4 (1:1000, Abcam, #ab137675), cadherin (1:1000, Abcam, #ab133168), vimentin (1:1000, Abcam, #ab8978), TAZ (1:1000, Abcam, #ab224239), complex III subunit core (CIII-core2, 1:1000, Invitrogen, #459220), complex II (CII-30, 1:1000, Abcam, #ab110410), complex IV subunit II (CIV-II, 1:1000, Abcam, #ab110268), Drp1 (1:1000, Abcam, #ab56788), Fis1 (1:1000, Abcam, #ab71498), Opa1 (1:1000, Abcam, #ab42364), Mfn1 (1:1000, Abcam, #ab57602), Mff (1:1000, Cell Signaling Technology, #86668), Bcl2 (1:1000, Cell Signaling Technology, #3498), Bax (1:1000, Cell Signaling Technology, #2772), caspase-9 (1:1000, Cell Signaling Technology, #9504), Bad (1:1000; Abcam; #ab90435), Tom20 (1:1000, Abcam, #ab186735), cyt-c (1:1000; Abcam; #ab90529), GAPDH (1:1000, Cell Signaling Technology, #5174), JNK (1:1000; Cell Signaling Technology, #4672), and p-JNK (1:1000; Cell Signaling Technology, #9251)]. After being washed with TBST, the membranes were incubated with the secondary antibodies for 45 min at room temperature. The bands were observed with an enhanced chemiluminescence (ECL) substrate kit (Beyotime, China, Cat. No. P0018F). The mean densities of the bands were represented as the optical density in units/mm^2^ and normalized to that of loading control (Quantity One, version 4.6.2; Bio-Rad Laboratories, Inc.)

### Immunofluorescence

Cells were washed with PBS at room temperature to remove the DMEM. Then, the cells were fixed in 3.7% paraformaldehyde for 30 min at room temperature and permeabilized with 0.1% Triton X-100 for 10 min at 4 °C. The cells were then washed with PBS, and 10% goat serum albumin was used to block the samples for 45 min at room temperature. The samples were again washed with PBS, and the primary antibodies [p-JNK (1:500; Cell Signaling Technology, #9251), cyt-c (1:500; Abcam; #ab90529), Drp1 (1:500, Abcam, #ab56788), CDK4 (1:500, Abcam, #ab137675), cyclin D1 (1:500, Abcam, #ab134175), and Tom20 (1:500, Abcam, #ab186735)] were added. The samples were incubated overnight at 4 °C. After being washed with PBS three times to remove the primary antibodies, the cells were incubated with the secondary antibodies for 45 min at room temperature [37]. After the cells were again washed with PBS to remove the free second antibodies and were loaded with DAPI, they were observed under an inverted microscope. Mitochondrial fission was observed via immunofluorescence using the Tom20 antibody. Images were captured, and the average length of the mitochondria was used to quantify the mitochondrial fission [38].

### Statistical analysis

All statistical analyses in the present study were performed in SPSS software (version 19.0). Our data are expressed as the mean ± SEM. Results for more than two groups were evaluated by one-way analysis of variance followed by Bonferroni’s multiple comparison test. A P value < 0.05 was considered significant.

## Results

### IL-2 promotes sorafenib-mediated apoptosis in HepG2 and Huh7 cells

First, sorafenib was added into the medium of liver cancer cell lines (HepG2 cells and Huh7 cells) to repress the cancer cell viability. Compared to the control group, the sorafenib treatment group displayed markedly reduced cell viability, as assessed via MTT assay (Fig. 1a, b), suggesting that sorafenib is cytotoxic to liver cancer cell lines. Similarly, the cell death rate, as evaluated by the LDH release assay, also increased in response to sorafenib treatment in both the HepG2 and the Huh7 cells (Fig. 1c, d). To explore whether the tumour-suppressive effect of sorafenib could be enhanced by combining sorafenib with IL-2-based therapy, different doses of IL-2 were added to the medium. As shown in Fig. 1a, b, the cell viability of both HepG2 cells and Huh7 cells progressively decreased with increasing IL-2 concentrations. IL-2 treatment also dose-dependently elevated the cell death index, as determined by the LDH release assay (Fig. 1c, d). Altogether, these results indicated that IL-2 supplementation augmented the anti-tumour effect of sorafenib in HepG2 and Huh7 cells. The minimum toxic concentration of IL-2 was 5 ng/ml; therefore, that dose was used in subsequent functional studies. To exclude the influence of IL-2/sorafenib co-treatment on normal hepatocytes, L02 normal liver cells were treated with IL-2 and sorafenib. As shown in Additional file 1: Figure S1, we found that neither IL-2 nor sorafenib treatment affected the viability of L02 cells, as assessed via MTT assay and LDH release assay. Subsequently, TUNEL staining was used to detect cell apoptosis after IL-2 and sorafenib co-treatment in HepG2 cells. As shown in Fig. 1e–g, the number of TUNEL-positive cells increased with sorafenib treatment and was further elevated in response to IL-2 administration in both HepG2 cells and Huh7 cells. Similarly, caspase-3 activity increased in response to sorafenib treatment, and this effect was enhanced by IL-2 treatment (Fig. 1h, i). In all, our data indicated that IL-2 supplementation augmented sorafenib-mediated cell apoptosis in both HepG2 cells and Huh7 cells.

**Fig. 1:** IL-2 treatment enhanced the pro-apoptotic effects of sorafenib. **a**, **b** Cell viability was measured via MTT assay in HepG2 cells and Huh7 cells. The different doses of IL-2 were added in the presence of 5 μM sorafenib. **c**, **d** Cell death was evaluated via LDH release assay in HepG2 cells and Huh7 cells. The different doses of IL-2 were added in the presence of 5 μM sorafenib. **e**–**g** A TUNEL assay was performed to observe the cell apoptotic rate. IL-2 (5 ng/ml) treatment was carried out in the presence of 5 μM sorafenib. **h**, **i** Caspase-3 activity was measured in HepG2 cells and Huh7 cells. IL-2 (5 ng/ml) treatment was carried out in the presence of 5 μM sorafenib. *P < 0.05 vs. control group; ^#^P < 0.05 vs. sorafenib group. *Cont* control

### IL-2 further repressed cell migration and proliferation in the presence of sorafenib

Cancer proliferation was observed via EdU assay. The results shown in Fig. 2a–c revealed that sorafenib attenuated the percentage of EdU^+^ cells regardless of whether they were HepG2 cells or Huh7 cells. Interestingly, the anti-proliferative capacity of sorafenib was strengthened by IL-2 treatment (Fig. 2a–c), suggesting that IL-2 in combination with sorafenib further disrupted cancer growth. Similar results were observed for the expression of proteins related to the cell cycle. Cyclin D1, PCNA and CDK4 were abundant in the control group and were reduced in response to sorafenib treatment (Fig. 2d–j). IL-2 administration caused a further decline in the expression of cyclin D1, PCNA and CDK4 in both HepG2 cells and Huh7 cells (Fig. 2d–j). Taken together, our data support a synergistic role for sorafenib and IL-2 in repressing the multiplication of cancer cells.

**Fig. 2:** IL-2 further repressed cell migration and proliferation in the presence of sorafenib. **a**–**c** An EdU assay was used to observe the proliferative cells. The number of EdU-positive cells was recorded. **d**–**j** Western blotting analysis for the proteins related to cell proliferation. IL-2 (5 ng/ml) treatment was carried out in the presence of 5 μM sorafenib. **k**–**m** A transwell assay was conducted to determine the cell migration in response to IL-2 and sorafenib co-treatment. **n**–**r** The proteins related to cell migration were analysed via western blotting. IL-2 (5 ng/ml) treatment was carried out in the presence of 5 μM sorafenib. *P < 0.05 vs. control group; ^#^P < 0.05 vs. sorafenib group. *Cont* control

To examine cell migration, a transwell assay was performed. The number of migrated cells was reduced by sorafenib treatment and was further depressed with IL-2 treatment (Fig. 2k–m). In addition, proteins related to cancer migration, such as cadherin and vimentin, were negatively regulated by sorafenib, and this effect was enhanced by IL-2 treatment in both HepG2 and Huh7 cells (Fig. 2n–r). In summary, the sorafenib-induced impairment of migration was strengthened by IL-2. Because no phenotypic differences were noted between HepG2 and Huh7 cells with regards to apoptosis, proliferation or migration, the HepG2 cell line was used for subsequent molecular experiments.

### IL-2 in combination with sorafenib interrupts mitochondrial metabolism

Cellular proliferation, migration and survival are heavily dependent on the production of sufficient energy by the mitochondria; thus, mitochondrial metabolism was monitored. Cellular ATP production was repressed by sorafenib in HepG2 cells, and this effect was reinforced by IL-2 supplementation (Fig. 3a). Mitochondrial energy production primarily relies on the activity of mitochondrial respiratory enzymes [20, 39], which convert the mitochondrial membrane potential into the chemical ATP. Interestingly, the expression levels of the mitochondrial respiratory proteins were downregulated by sorafenib (Fig. 3b–e); this tendency was exacerbated by IL-2 treatment. In addition, the mitochondrial potential, as assessed by JC-1 staining, was also negatively regulated by sorafenib (Fig. 3f–g). IL-2 treatment further repressed the mitochondrial potential, as evidenced by a lower ratio of red/green fluorescence intensity.

**Fig. 3:** IL-2 and sorafenib co-treatment inhibited mitochondrial energy metabolism. **a** ATP production was measured in HepG2 cells subjected to IL-2 and sorafenib co-treatment. **b**–**e** Mitochondrial respiratory proteins were analysed via western blotting in HepG2 cells. IL-2 (5 ng/ml) treatment was carried out in the presence of 5 μM sorafenib. **f**, **g** Mitochondrial potential was detected through JC-1 staining. Red fluorescence, which indicated normal mitochondrial potential, was converted into green fluorescence after a reduction in mitochondrial potential. **h**, **i** The remaining glucose and the produced LDH in the medium were analysed for HepG2 cells. IL-2 (5 ng/ml) treatment was carried out in the presence of 5 μM sorafenib. *P < 0.05 vs. control group; ^#^P < 0.05 vs. sorafenib group. *Cont* control

Finally, we measured the amount of glucose remaining in the medium to directly evaluate the cellular mitochondrial metabolism. Compared to the control group, the sorafenib treatment group showed reduced glucose uptake from the medium (Fig. 3h). Lactate production was also reduced in response to sorafenib treatment (Fig. 3j). IL-2 supplementation further repressed glucose absorption and lactate generation (Fig. 3h–j), indicating the cessation of glucose absorption, consumption and metabolism, possibly due to mitochondrial dysfunction. Altogether, our data highlight a causal relationship between IL-2 administration and mitochondrial dysfunction when sorafenib is present.

### IL-2 induces mitochondrial apoptosis in sorafenib-treated cells

Given the links between IL-2 and mitochondrial dysfunction, we tested whether IL-2 would amplify sorafenib-activated mitochondrial apoptosis in HepG2 cells. As shown in Fig. 4a, b, mitochondrial ROS production, an early molecular event in mitochondrial apoptosis, increased significantly in response to sorafenib treatment in HepG2 cells, and ROS generation was further evoked by IL-2 (Fig. 4a, b). The sorafenib-mediated ROS production was closely associated with a drop in the concentration of antioxidants such as GSH, SOD and GPX (Fig. 4c–e). IL-2 treatment contributed to a further loss of these antioxidants, suggesting a permissive role for IL-2 in cancer oxidative stress.

**Fig. 4:** IL-2 activated the mitochondrial apoptotic pathway in the presence of sorafenib. **a**, **b** Mitochondrial ROS production was detected in HepG2 cells. IL-2 (5 ng/ml) treatment was carried out in the presence of 5 μM sorafenib. **c**–**e** The antioxidants in HepG2 cells under IL-2 and sorafenib co-treatment were measured via ELISA. **f** The mPTP opening rate was analysed to determine the mitochondrial damage. IL-2 (5 ng/ml) treatment was carried out in the presence of 5 μM sorafenib. **g**, **h** Cyt-c liberation was observed via immunofluorescence. **i**–**o** Mitochondrial apoptotic proteins were analysed by western blotting. The sorafenib-mediated upregulation of apoptotic proteins was further augmented by IL-2 treatment. *P < 0.05 vs. control group; ^#^P < 0.05 vs. sorafenib group. *Cont* control

A late molecular feature of mitochondrial damage is the opening of the mitochondrial permeability transition pore (mPTP), a channel necessary to enable the transmission of mitochondrial pro-apoptotic factors into the cytoplasm/nucleus [40, 41]. Sorafenib-mediated mPTP opening was enhanced by IL-2 in HepG2 cells (Fig. 4f). We also found through immunofluorescence assay that cyt-c, a type of mitochondrial pro-apoptotic protein, was released into the nucleus upon sorafenib treatment due to the prolonged open state of the mPTP (Fig. 4g, h). IL-2 treatment facilitated the cyt-c translocation, as determined by analysis of the fluorescence intensity of cyt-c in the nucleus (Fig. 4g, h). This finding was also validated via western blotting. The level of mitochondrial cyt-c declined in sorafenib-treated cells; this decrease was accompanied by an increase in the expression of cytoplasmic cyt-c (Fig. 4i, j), an effect that was enhanced by IL-2. We also found that mitochondrial apoptotic proteins such as Bad, Bax and caspase-9 were all upregulated by sorafenib treatment (Fig. 4i–o). This upregulation was followed by a fall in the content of anti-apoptotic factors (Fig. 4i–o). The sorafenib-initiated mitochondrial apoptosis was amplified by IL-2 (Fig. 4i–o). Taken together, our data illustrate that IL-2 can promote sorafenib-mediated mitochondrial apoptosis in HepG2 cells.

### Mitochondrial fission is augmented by IL-2 in the presence of sorafenib

To explain the additional action of IL-2 in activating mitochondrial apoptosis in the presence of sorafenib, we focused on mitochondrial fission, which is the upstream trigger of mitochondrial apoptosis through multiple biological processes [19, 20]. Mitochondrial fission was first examined by western blotting. Mitochondrial fission-related proteins such as Drp1, Fis1 and Mff [42] were slightly upregulated in sorafenib-treated cells (Fig. 5a–f) and were highly elevated in response to IL-2 supplementation. These data indicate that mitochondrial fission seems to be initiated by sorafenib and is further amplified by IL-2 supplementation. In addition, we examined the proteins related to mitochondrial fusion, the defensive system used to correct excessive mitochondrial division. Compared to those in the control group, the levels of mitochondrial fusion-related proteins, such as Mfn1 and Opa1, were marginally downregulated in the sorafenib-treated group (Fig. 5a–f), and this effect was exaggerated by IL-2. These data suggest that IL-2 helps sorafenib to hinder the mitochondrial fusion system, indirectly promoting mitochondrial fission.

**Fig. 5:** IL-2 enhanced sorafenib-initiated mitochondrial fission. **a**–**f** Western blotting was used to analyse the proteins related to mitochondrial fusion and mitochondrial fission. Drp1, Fis1 and Mff are factors involved in mitochondrial fission. In contrast, mitochondrial fusion is regulated by Mfn1 and Opa1. IL-2 and sorafenib co-treatment elevated the mitochondrial fission proteins and repressed the mitochondrial fusion factors. **g**, **h** Mitochondrial fission was observed via immunofluorescence using the Tom20 antibody. Then, the average length of mitochondria was measured in HepG2 cells. *P < 0.05 vs. control group; ^#^P < 0.05 vs. sorafenib group. *Cont* control

Subsequently, an immunofluorescence assay for mitochondria was conducted to observe the mitochondrial fission. In sorafenib-treated cells, the mitochondrial network divided into several fragmented mitochondria in response to mitochondrial fission (Fig. 5g). This alteration was more prominent in IL-2-challenged cells. We further measured the average length of the mitochondria to quantify the mitochondrial fission. The average length of the mitochondria was reduced to some extent under sorafenib treatment (Fig. 5h), and this effect was augmented by IL-2. Overall, we confirmed that IL-2 promotes sorafenib-triggered mitochondrial fission in HepG2 cells.

### IL-2 regulates mitochondrial fission via the JNK-TAZ pathways

The mechanism by which IL-2 boosts mitochondrial fission in the presence of sorafenib was unclear. Since JNK and TAZ have been well documented as activators of mitochondrial fission, we wondered whether JNK-TAZ pathways were also involved in IL-2-exacerbated mitochondrial fission in the presence of sorafenib. Western blotting analysis revealed that both JNK phosphorylation and TAZ expression were slightly increased in response to sorafenib treatment (Fig. 6a–c) and were considerably upregulated with IL-2 supplementation. These findings suggest that the JNK-TAZ pathways are regulated by IL-2 and sorafenib co-treatment.

**Fig. 6:** IL-2 and sorafenib co-treatment regulated mitochondrial fission via the JNK-TAZ pathways. **a**–**c** JNK phosphorylation and TAZ expression were measured via western blotting. SP600125, an inhibitor of JNK, was used to inhibit the activity of the JNK-TAZ pathways. **d**, **e** Mitochondrial fission was observed via immunofluorescence, and the average length of the mitochondria was recorded. **f**–**h** The regulatory effects of IL-2 and sorafenib co-treatment on the JNK-TAZ pathways and mitochondrial fission were monitored via immunofluorescence. IL-2 and sorafenib co-treatment promoted the upregulation of JNK phosphorylation, which was accompanied by an increase in Drp1, a factor for mitochondrial fission. *P < 0.05 vs. control group; ^@^P < 0.05 vs. IL-2+ sorafenib group. *Cont* control

To demonstrate whether the JNK-TAZ pathways were required to initiate mitochondrial fission, we inhibited JNK activity with a pathway blocker, SP600125. The inhibitory efficiency was validated via western blotting as shown in Fig. 6a–c. After blockade of JNK, the mitochondrial fission was monitored by immunofluorescence as described previously. Compared to the fragmented mitochondria under IL-2 and sorafenib co-treatment, the mitochondria of SP600125-treated cells maintained an interconnected phenotype (Fig. 6d). Similarly, the average length of the mitochondria was increased after SP600125 treatment when compared to the average length after IL-2 and sorafenib co-treatment (Fig. 6e). We also measured the alteration of mitochondrial fission-related proteins, such as Drp1, through co-immunofluorescence. The fluorescence intensity of Drp1 closely paralleled the content of p-JNK upon IL-2 and sorafenib co-treatment (Fig. 6f–h); higher p-JNK expression was accompanied by increased Drp1 fluorescence intensity. However, inhibition of JNK abrogated the stimulatory effect of IL-2/sorafenib on Drp1 expression (Fig. 6f–h). Collectively, the above data verify the necessity of the JNK-TAZ pathways in IL-2/sorafenib-mediated mitochondrial fission.

### JNK-TAZ pathways are also involved in IL-2-mediated migration inhibition and proliferation arrest

Finally, we wanted to know whether the JNK-TAZ pathways also participate in the migration and proliferation of HepG2 cells. An immunofluorescence assay for cell cycle proteins confirmed that IL-2/sorafenib promoted the expression of CDK4 and cyclin D1 (Fig. 7a–c), and this effect was negated by blocking the JNK-TAZ pathways. In addition, the EdU assay also illustrated that IL-2/sorafenib co-treatment attenuated the ratio of EdU-positive cells by activating the JNK-TAZ pathways (Fig. 7d, e). These data indicate that IL-2/sorafenib-modulated cancer proliferation is dependent on the activity of the JNK-TAZ pathways.

**Fig. 7:** Cell migration and proliferation were also regulated by IL-2/sorafenib co-treatment through the JNK-TAZ pathways. **a**–**c** Immunofluorescence assay for cell proliferation-related factors. IL-2/sorafenib co-treatment elevated the expression of CDK4 and cyclin D1, which was repressed by SP600125, an inhibitor of the JNK-TAZ pathways. **d**, **e** An EdU assay was performed to quantify the cell proliferation. The number of EdU-positive cells was recorded. **f**–**h** Cell migration factors such as CXCR4 and CXCR7 were measured via western blotting. *P < 0.05 vs. control group; ^@^P < 0.05 vs. IL-2+ sorafenib group. *Cont* control

With respect to cancer migration, molecular regulators, such as CXCR4 and CXCR7, were reduced by IL-2/sorafenib co-treatment and were reversed to near-normal levels after the inactivation of the JNK-TAZ pathways (Fig. 7f–h). These data illustrate the critical role played by the JNK-TAZ pathways in cancer migration.

## Discussion

Despite advances in the molecular understanding of HCC, few effective drugs are available in clinical practice to prevent its development. Sorafenib, a first-line targeted therapy drug, has shown a significant survival benefit for patients with HCC in global multiple-centre clinical trials [43, 44]. However, its efficacy is limited to a 3-month extension in survival time [45, 46]. Although several attempts have been made to elucidate the resistance mechanism of HCC against sorafenib, no solid conclusions have been drawn [47]. Several studies have suggested that the alteration of glucose metabolism and/or the downregulation of the Raf-1 kinase inhibitory protein could be possible resistance mechanisms in patients receiving sorafenib [48, 49]. In the present study, our data suggest an option to enhance the therapeutic efficacy of sorafenib in killing liver cancer cells. A combination of sorafenib and IL-2 reduced the viability of liver cancer cell lines in vitro compared to the viability after sorafenib treatment alone. Moreover, cancer cell migration and proliferation were also repressed by sorafenib in conjunction with IL-2. At the molecular level, IL-2 supplementation assisted sorafenib in inducing mitochondrial injury by activating fatal mitochondrial fission. We also demonstrated that IL-2, in the presence of sorafenib, modified mitochondrial fission via the JNK-TAZ pathways. This is the first investigation to present a novel way to enhance the anti-tumour effect of sorafenib on liver cancer in vitro. Our findings will pave the way for new treatment modalities to control HCC progression by optimizing sorafenib-based therapy.

In the present study, we demonstrated that IL-2 facilitated the pro-apoptotic effects of sorafenib by augmenting mitochondrial fission. Mitochondrial fission is a physical process that modulates the quantity and quality of mitochondrial mass [50]. Moderate mitochondrial fission is necessary for cellular metabolism through the timely production of daughter mitochondria [51]. Moreover, mitochondrial fission helps mitochondria to remove damaged parts, thus enabling mitochondrial turnover and renewal [52]. However, excessive mitochondrial fission converts the mitochondrial network into discontinuous debris, leading to mitochondrial dysfunction. Previous studies on cardiac ischemia/reperfusion have demonstrated that mitochondrial fission activates mitochondrial apoptosis via the HK2-VDAC1-mPTP pathway and the mROS/cardiolipin/cyt-c axis [42]. More recent studies on pancreatic cancer have also found that cancer cell proliferation, migration and survival are closely regulated by mitochondrial fission [21]. Similar findings have been reported for colorectal cancer [53], endometriosis [22], and liver cancer [25]. Consistent with these reports, our data also identify mitochondrial fission as the critical upstream signal for mitochondrial homeostasis in liver cancer cells.

We also demonstrated in this study that mitochondrial fission is drastically activated by IL-2 in the presence of sorafenib, and this regulatory mechanism is dependent on the JNK-TAZ pathways. Notably, no studies investigating the detailed role of IL-2 in mitochondrial fission have yet been conducted. Thus, our investigation provides the first evidence that the tumour-suppressive effects of IL-2 on liver cancer may be attributable to the activation of mitochondrial fission. Notably, the apoptotic rate of HepG2 cells was progressively increased with a rise in the dose of IL-2. The minimum toxic concentration of IL-2 was 5 ng/ml, and therefore, this dose was used to explore whether IL-2 could augment the efficiency of sorafenib-based therapy. Subsequently, we demonstrated that IL-2 regulates mitochondrial fission via the JNK-TAZ pathways. Previous studies have reported the critical role of JNK and TAZ in activating mitochondrial fission in several disease models. For example, in human rectal cancer cells, activation of the JNK pathway promotes mitochondrial fission, thereby reducing cancer cell survival and migration [53]. In primary hepatocytes, the inhibition of mitochondrial fission through the modulation of JNK protects the cells against senecionine-induced mitochondrial apoptosis [54]. In breast cancer cells, disruption of the JNK pathway inhibits mitochondrial fission and represses cancer cell proliferation and survival [55]. The above information lays a foundation to help us understand the role of JNK in regulating mitochondrial fission. With respect to TAZ, an early study revealed that mitochondrial fission could be controlled by TAZ through the regulation of mitochondrial lipid synthesis [56]. Subsequent experiments verified that breast cancer migration is highly controlled by TAZ through mitochondrial fission [57]. Furthermore, TAZ has been found to promote mitochondrial fission and induce stem cell differentiation [58]. Such results describe the causal relationship between TAZ and mitochondrial fission. Similar to these findings, our study revealed that the JNK-TAZ pathways are activated by IL-2 in the presence of sorafenib and contribute to mitochondrial fission, ultimately repressing liver cancer cell survival, migration and proliferation. These findings inform us of the anti-tumour molecular mechanisms activated by IL-2 in combination with sorafenib and suggest that strategies targeting mitochondrial fission and the JNK-TAZ axis would yield additional clinical benefits for patients suffering from HCC. To the end, we also found that the survival rate and proliferative index of HepG2 cells were still high in response to IL-2/sorafenib co-treatment. Accordingly, more attempts are required to further enhance the sensitivity of HCC to sorafenib-based therapy. Although we observed the inhibitory effect of IL-2/sorafenib co-treatment on HepG2 cell migration, the IL-2/sorafenib-mediated cell apoptosis and proliferation arrest may also influence the HepG2 cell migration. Further investigation of the direct role of IL-2/sorafenib co-treatment in HCC migration is required.

## Conclusions

Taken together, our data indicate that additional supplementation with IL-2 can enhance the tumour-killing activity of sorafenib. IL-2 in combination with sorafenib repressed liver cancer cell proliferation, migration and survival by promoting mitochondrial dysfunction. The synergetic effects of IL-2 and sorafenib were primarily dependent on mitochondrial fission through the activation of the JNK-TAZ pathways. These findings provide new insights into the mechanisms of these drugs and suggest novel strategies to induce cancer cell death with sorafenib therapy.

## Additional file

**Additional file 1: Figure S1.** The influence of IL-2 and sorafenib treatment on the viability of L02 normal liver cells. A. MTT assay was used to evaluate the cell viability. B. LDH release assay was performed to detect the cell death in response to Il-2 and sorafenib treatment.

## Abbreviations

TAZ: transcriptional co-activator with PDZ-binding motif
Cyt-c: cytochrome c
mPTP: mitochondrial permeability transition pore
IL-2: interleukin-2
HCC: hepatocellular carcinoma
